The article "English Text Readability Measurement Based on Convolutional Neural Network: A Hybrid Network Model" was published in 2022. Journal: Comput Intell Neurosci.

# English Text Readability Measurement Based on Convolutional Neural Network: A Hybrid Network Model

**DOI:** 10.1155/2022/6984586

**Published:** 2022-03-15

**Authors:** Lihua Jian, Huiqun Xiang, Guobin Le

**Affiliations:** ^1^School of International Education, Hunan University of Medicine, Hunan, Huaihua 418000, China; ^2^Changsha Vocational and Technical College, Hunan, Changsha 410200, China; ^3^School of Foreign Languages, Huaihua University, Huaihua 418000, China

## Abstract

Text readability is very important in meeting people's information needs. With the explosive growth of modern information, the measurement demand of text readability is increasing. In view of the text structure of words, sentences, and texts, a hybrid network model based on convolutional neural network is proposed to measure the readability of English texts. The traditional method of English text readability measurement relies too much on the experience of artificial experts to extract features, which limits its practicability. With the increasing variety and quantity of text readability measurement features to be extracted, it is more and more difficult to extract deep features manually, and it is easy to introduce irrelevant features or redundant features, resulting in the decline of model performance. This paper introduces the concept of hybrid network model in deep learning; constructs a hybrid network model suitable for English text readability measurement by combining convolutional neural network, bidirectional long short-term memory network, and attention mechanism network; and replaces manual automatic feature extraction by machine learning, which greatly improves the measurement efficiency and performance of text readability.

## 1. Introduction

As long as people create, study, share, and disseminate ideas through written language, the concept of text difficulty will be always an important aspect of people's communication and education [1–3]. More than 2000 years ago, ancient Athenian scholars paid attention to the difficulty of reading the text and pointed out that students studying law usually face the problem that their laws are difficult to be understood by the audience. If the audience does not understand them, they cannot understand and support the truth they say in the legal debate. In order to better explain the meaning of the law to the audience, language rhetoric training has become an important part of learning law. In the process of language learning, improving reading ability is also an important part of language acquisition, and its reading comprehension ability is also the key standard to evaluate learners' language skills [2]. The most effective way to improve reading comprehension is to provide learners with reading materials slightly higher than their reading ability. Reading too simple text is meaningless repetitive work. If the text is too difficult, language learners will lose their confidence and interest in learning the language.

Therefore, classifying reading materials through the reading ability of learners or audiences plays a vital role in foreign language learning [3, 4]. This task of sorting out reading learning materials according to the reading difficulty of the text is called text readability measurement or text reading difficulty evaluation, which is an important natural language processing (NLP) problem [5–8]. Since the last century, there has been a systematic and scientific method for understanding the subjective and objective factors related to text readability, better supporting readers to understand more difficult texts, or correctly finding the task of text reading difficulty. Based on the research of these systems, text readability has been defined as the sum of all elements that affect readers' understanding of text materials, reading speed, and interest in text content. These elements may include the complexity of text syntax, the semantic familiarity of readers with some concepts in the text, whether there are supporting graphics or illustrations to explain the text, the complexity of logical argument or inference used to connect various views in the text, and many other important contents [9–11]. In addition to these text features, readers' own characteristics, that is, their education, social background, interests, professional knowledge, learning motivation, and other factors, can play a key role in the readability of the text.

In view of the importance of text readability in meeting people's information needs and the explosive growth of modern information, the measurement demand of text readability is increasing, and the influence of effective text readability evaluation is also increasing day by day [12]. The so-called effectively quantifying the reading difficulty of a text means that the reading difficulty level of the corresponding text is expressed by using the text as input and in the form of prediction such as estimated digital score or difficulty level category label, or used to indicate the reading level and understanding ability of a given population to the corresponding text [13–17]. In this paper, we focus on the internal language feature factors affecting text readability, such as semantics and syntax, but do not pay attention to the external feature factors affecting text reading difficulty, such as font size or font color contrast, which affect readers' visual decoding ability, as well as readers' educational background, interests, and hobbies and other factors related to readers themselves.

The significance of this paper lies in the following points.

1. Automatic and effective measurement of text readability can liberate the unnecessary labor of some people, such as teachers, students, and web text processors, in finding and classifying the reading difficulty of relevant texts
2. Automatic and effective measurement of text readability is of great significance for the accessibility of key information and also plays a key role in specific application fields

The functions of readability measurement include the following: (1) It can provide language learners with extracurricular reading materials of different levels of difficulty suitable for their reading abilities at different stages, such as graded reading. (2) It can provide language teachers with teaching resources suitable for the difficulty of reading and provide guidance for their application of compiling teaching materials and test questions. (3) It can automatically calibrate and simplify public and private health information so that the public and patients can read and understand medical related text resources such as medical instructions, health questionnaires, and brochures. (4) It can provide suggestions for businesses to make effective product guides and other text documents for the public. (5) It can also be further applied to the accurate retrieval and recommendation of web text.

## 2. Related Works

The measurement of text readability usually refers to determining the difficulty of text content being understood by people [16, 17]. Generally, the readability of a text can be measured by a predefined readability level or readability score. In this paper, the readability level is used to measure the readability of text. The measurement of text readability can be regarded as a classification problem, that is, how to learn the prediction model according to the text set with determined readability level and then use the model to predict the text with unknown readability level.

The research on text readability measurement has a history of at least one century. However, this is far from a “solved” problem, and the automatic measurement of text readability is still a challenging research field. The research on the measurement of readability can be traced back to the 1920s. Early readability studies mainly focused on the lexical factors of the text and used proxy variables to represent the relevant characteristics of vocabulary, such as the difficulty, diversity, and scope of use. Whether one vocabulary difficulty standard is better than the other depends mainly on the experience of expert judges and correlation analysis. These works showed that the research on text readability began to pay attention to all aspects of feature selection. From 1940s to 1990s, the readability research system was initially formed. During this period, researchers continued to try various readability formulas, introduce proxy variables of lexical and syntactic information into the formulas, and make linear combinations, hoping to accurately evaluate the text readability and obtain an optimal reading difficulty measurement standard [18–20].

From 1980s to 1990s, researchers began to pay attention to the structural information of text and introduced cognitive theories such as connection theory, conceptual schema theory, prototype theory, and diffusion activation theory into the field of text readability to explain the way people store and retrieve information in long-term memory. Through human cognitive style, the concept of text readability is associated with text structure, and the characteristics of text organization structure, discourse coherence, and cohesion are introduced [21]. At the same time, we also pay attention to the measurement of lexical features, introduce statistical language model to statistically analyze the words and word occurrence order in a given text set, count the occurrence frequency of different words or word combinations in the text set, and use this probability to measure the difficulty of vocabulary reading.

Statistical language model is applied to measure the readability of science and technology web pages [22]. After that, with the development of natural language processing technology, such as part-of-speech tagging, syntax analysis, and language model, researchers can more deeply mine the content and structure of text, which makes the research of readability have new progress. Then, new text features are constantly explored, and new theories such as information theory have also been applied in the study of readability. At the same time, some new technologies in the field of machine learning, such as classification, regression, and sorting, are also used to design new readability evaluation methods, which gives birth to a new measurement method of text readability, that is, the text readability measurement method based on machine learning and complex features [23, 24].

Since the beginning of the twenty-first century, the text readability measurement method based on machine learning and complex features has continuously integrated various rich features and introduced various powerful machine learning frameworks to constantly refresh the performance of the text readability measurement model, which is still developing [24].

With the explosive growth of big data and the emergence of deep learning, a new measurement method has been introduced into the measurement of text readability. The text readability measurement method based on deep learning shows great advantages in measuring the accuracy and automation of text readability [25]. Therefore, this method is a new research trend of text readability measurement methods recently.

However, the research on the measurement of text readability mainly faces several challenges. Firstly, the traditional readability measurement, including readability formula method and measurement method based on artificial intelligence, heavily depends on the extraction of expert artificial features, which seriously lags behind the automation of readability measurement. In the era of big data, how to liberate a large number of labor forces and automatically extract features is a research difficulty. Secondly, with the development of natural language processing and machine learning technology, there are many manually extractable features (e.g., semantic and syntactic structure) that affect the difficulty of text reading. It is more and more difficult to manually extract new features. How to more comprehensively represent the features of text without introducing redundant features is also a difficulty. Thirdly, the measurement of text readability is oriented to different language learners, such as native English (L1) learners and nonnative English (L2) learners. However, the existing model method is difficult to use the same model method to measure the text reading difficulty of L1 and L2. A method that achieves good performance in L1 text readability does not necessarily have the same performance in L2 text.

## 3. English Text Readability Measurement Based on Convolutional Neural Network

With the rapid development of information technology, it is an era of knowledge explosion and tons of data growth. Finding text materials suitable for the required reading difficulty level in a large number of texts is a very time- and labor-consuming task for readers, which virtually increases their burden. Therefore, effectively measuring the readability of the text and providing readers with intuitive selection criteria will directly affect readers' reading efficiency, which is very necessary. Starting from the various challenges and difficulties faced by the current text readability measurement, this paper regards the text readability measurement task as a classification task and proposes a hybrid network model to measure English text readability based on convolutional neural network (CNN).

The traditional text readability measurement method has some fatal pain points. In the research process of text readability measurement, feature selection excessively depends on human experts, which limits the development of text readability measurement. There are a wide variety and a large number of existing features that measure text readability. It is more and more difficult to extract new features manually to improve the readability measurement performance, and even introduce redundant and irrelevant features to affect the readability measurement performance.

### 3.1. CNN Model Introduction

CNN [26] and long short-term memory network (LSTM) [27] are mature and successful deep learning models in the field of natural language processing. Now, these two network models are still the deep learning models that researchers focus on in various natural language related tasks. It is generally believed that CNN is good at capturing local features of language, while LSTM is good at processing sequence data and capturing long-distance dependent information.

In recent years, in order to integrate the advantages of CNN and LSTM, many studies have proposed a hybrid network model based on CNN and LSTM to solve the tasks related to natural language processing.

In order to capture the context information and local features of text, Peng et al. [28] used BiLSTM-DCNN hybrid network model to achieve good performance in text classification task. Fu et al. [29] used CNN-BiLSTM hybrid network model for beautiful sentence recognition. Through experimental comparison with CNN and BiLSTM networks, the results show that the hybrid network model can achieve higher accuracy. Hao et al. [2] also used CNN-BiLSTM hybrid network model to solve the task of Chinese text readability measurement and achieved good performance. For the task of measuring English text readability in this paper, we also use transfer learning and adopt the hybrid network model of CNN and BiLSTM to solve our research problem. CNN is good at extracting local features such as phrases, while BiLSTM can extract text context information and long-distance dependence information. The purpose of constructing this model is to make use of these two advantages [30, 31].

### 3.2. CNN Model

The structure of CNN model for English text readability measurement is shown in Figure 1.

#### 3.2.1. Word Vector Query Layer

The first layer is the word vector query layer, which is used to mathematically symbolize the natural language sequence to be processed; that is, each given word is projected into the word vector space to facilitate further processing in subsequent layers. The input to this layer is a series of words:

(1) $$\begin{array}{c} {\text{Input}}_{\text{layer}1}=\left[w_{1},w_{2},\ldots ,w_{M}\right]. \end{array}$$

The output of the query layer is the distributed vector representation of the words queried from GloVe word vector:

(2) $$\begin{array}{c} \bar{x}=\left[x_{1},x_{2},\ldots ,x_{n}\right], \end{array}$$

where *x*_*i*_ ∈ *R*^*d*^ and *n* is the length of the sequence.

#### 3.2.2. Convolution Layer and Max-Pooling Layer

Once the word vector representation $\bar{x}$ of the input sequence is queried, in order to more comprehensively extract local features from the sequence, the convolution layer will use multiple filters of different sizes to continuously perform convolution operation on the word vector sequence $\bar{x}$ by sliding.

If the filter size of the convolution layer is *k*, the filter can be expressed as a matrix:

(3) $$\begin{array}{c} m\in R^{k\times d}. \end{array}$$

In the filter sliding process, for each position *i* in the sequence, there is a window matrix ${\bar{w}}_{i}$ with *k* consecutive words, expressed as

(4) $$\begin{array}{c} {\bar{w}}_{i}=\left[x_{i},x_{i+1},\ldots ,x_{i+k-1}\right]. \end{array}$$

The filter matrix *m* is convoluted with the word window matrix ${\bar{w}}_{i}$ (k-gram) at each position in an effective way to generate a feature map:

(5) $$\begin{array}{c} c\in R^{L-k+1} \end{array}$$

The feature mapping of the word window vector $\bar{w}$ at position *i* can be calculated as

(6) $$\begin{array}{c} c_{i}=\sigma \left(\bar{w}⊗m+b\right), \end{array}$$

where ⊗ is multiplication, *b* is bias, and *σ* is the activation function of sigmoid.

Then, in the convolution layer, the max pooling will be further used for the results of convolution calculation. The max pooling will filter the maximum value in *c*_*i*_ as the feature of the filter corresponding to the *i*th word. The max pooling can reduce the output parameters of CNN and the risk of overfitting and also reduce the impact of filling 0 when processing input sequences of equal length.

In terms of convolution operation mode, convolution layer is similar to *n*-gram language model. It is good at extracting local context information in article sequence, so as to improve the performance of the model.

#### 3.2.3. Circulation Layer

After generating the embedding (whether from the convolution layer or directly from the query layer), the loop layer starts processing the input sequence to generate a representation of a given article. Ideally, the representation can encode all the information needed to measure text readability. However, because the text is usually very long and consists of hundreds of word sequences, the vector representation learned by the final state of the loop layer may not be enough for accurate readability measurement.

For this reason, we keep all the intermediate states of the loop layer so that we can track and process the important information of the article. For the circular layer, based on the experimental experience, we choose BiLSTM to extract the long-distance dependence information of text context and sequence.

In order to control the information flow during the processing of the input sequence, the LSTM uses three gates to forget or remember the transmitted information of the sequence. The functions of LSTM are described as follows:

(7) $$\begin{array}{c} i_{t}=\sigma \left(W_{i}\cdot X_{t}+U_{i}\cdot h_{t-1}+b_{i}\right),\\ f_{t}=\sigma \left(W_{f}\cdot X_{t}+U_{f}\cdot h_{t-1}+b_{f}\right),\\ {\tilde{c}}_{t}=\tanh\left(W_{c}\cdot X_{t}+U_{c}\cdot h_{t-1}+b_{c}\right),\\ c_{t}=i_{t}\circ {\tilde{c}}_{t}+f_{t}\circ c_{t-1},\\ o_{t}=\sigma \left(W_{o}\cdot X_{t}+U_{o}\cdot h_{t-1}+b_{o}\right),\\ h_{t}=o_{t}\circ \;\tanh\left(c_{t}\right)\text{,} \end{array}$$

where *X*_*t*_ and *h*_*t*_ are the input and output vectors at time *t*, respectively; *W*_*i*_, *W*_*f*_, *W*_*c*_, *W*_*o*_, *U*_*i*_, *U*_*f*_, *U*_*c*_, *U*_*o*_ are weight matrices; *b*_*i*_, *b*_*f*_, *b*_*c*_, *b*_*o*_ are bias vectors; and the symbol ∘ represents element-by-element multiplication.

#### 3.2.4. ATT/MoT Pooling Layer

This layer is connected behind the circulating layer and receives the output *H*=(*h*_1_, *h*_2_ …, *h*_*M*_) of the circulating layer. It is responsible for aggregating the variable length input H into a fixed length vector, so as to facilitate the use of subsequent network layers. There are generally two common methods for this layer, mean over time and attention pooling.

*(1) Mean over time method*. The average time layer receives *M* vectors with dimension *d*_*r*_ as input and calculates average vectors of the same length. The calculation formula is defined as follows:

(8) $$\begin{array}{c} v=\frac{\sum_{i=1}^{M}h_{i}}{M}. \end{array}$$

After the vector is calculated, it is sent to the subsequent network layer for corresponding operation.

*(2) Attention-pooling method*. The average time layer is equivalent to assigning an equal weight 1/*M* to the output *H* of the cycle layer, and the average time layer can also be replaced by a self-attention mechanism. The self-attention mechanism can learn the importance of the output of each intermediate state of the loop layer to the characterization of the whole document and assign a weight *α*_*i*_ to each output state *h*_*i*_. The calculation formula is defined as follows:

(9) $$\begin{array}{c} u=\tanh\left(Wh_{i}+b\right),\\ \alpha_{i}=\frac{\exp\left(u^{T}u_{w}\right)}{\sum_{i}\exp\left(u^{T}u_{w}\right)},\\ v=\sum_{i}\alpha_{i}h_{i}\text{,} \end{array}$$

where *h*_*i*_ represents the output of the intermediate state of the loop layer and *u*_*w*_ represents the vector representing the text context information. This vector is an initialization vector and will be automatically learned in the backpropagation.

#### 3.2.5. Softmax Layer

The final representation vector *v* of the text is obtained from the previous pooling layer and then sent to the softmax layer for classification. In this CNN model, cross entropy is selected as the loss function.

## 4. Case Study

### 4.1. Data Set

The existing gold data sets for English text readability measurement are Weekly Reader data set and WeeBit data set. In particular, WeeBit data set is one of the most popular data sets in text readability measurement tasks, with the largest amount of data and the most standard readability label [32].

WeeBit data set consists of two parts of data. The first part is Weekly Reader corpus, which is also one of the popular gold data sets in English text readability measurement tasks. The corpus comes from Weekly Reader (https://www.weeklyreader.com), an American educational news magazine. The texts in the magazine are compiled by educational experts according to the readers' age, and their age groups are designated as the reading difficulty level of the corresponding texts. The text content of the magazine is mainly applicable to the reading objects at ages 7-8, 8-9, 9-10, and 10–12. Another part of the data comes from the BBC Bitesize website, which provides readers of different ages with articles of corresponding difficulty. The WeeBit corpus uses text data corresponding to reading difficulty from two age groups on the BBC Bitesize website, which are 11–14 years old and 14–16 years old, respectively. These two parts of data are combined to form WeeBit corpus.

Because these two data sets are popular and authoritative in the field of English text readability measurement and in order to better compare our experimental results with existing methods, we use these two data sets. The details of these two data sets are shown in Table 1.

### 4.2. Evaluating Indicator

This paper uses the two most commonly used evaluation indicators in text readability measurement tasks, accuracy and Pearson correlation.

#### 4.2.1. Accuracy

In this paper, ACC is used to express the accuracy. We suppose that there are two types of original samples: P positive samples in total, marked as 1; N negative samples, marked as 0. After classification, TP samples with category 1 are correctly determined as 1 by the model, and FN samples with category 1 are determined as 0 by the model. Obviously, *P* = TP + FN. FP samples with category 0 are correctly determined as 1 by the model, and TN samples with category 0 are determined as 0 by the model. Obviously, *N* = FP + TN. Then, ACC can be defined as follows:

(10) $$\begin{array}{c} \text{ACC}=\frac{\text{TP}+\text{TN}}{P+N}. \end{array}$$

Accuracy (ACC) reflects the classifier's ability to classify the whole sample, that is, the ability to classify positive samples as positive and negative samples as negative.

#### 4.2.2. Pearson correlation

In this paper, PCC is used to express the Pearson correlation. PCC is defined as the quotient of covariance and standard deviation between two sequence variables, which is as follows:

(11) $$\begin{array}{c} \text{PCC}\left(X,Y\right)=\frac{E\left(\text{XY}\right)-E\left(X\right)E\left(Y\right)}{\sqrt{E\left(X^{2}\right)-E^{2}\left(X\right)}\sqrt{E\left(Y^{2}\right)-E^{2}\left(Y\right)}}. \end{array}$$

PCC can describe the correlation between two sequences *X* and *Y*, and the value range of PCC is [−1, 1]. When PCC > *O*, *X* and *Y* are positively correlated. When PCC <0, *X* and *Y* are negatively correlated. When PCC = 0, the two variables are not related. Generally, the greater the absolute value of PCC, the stronger the correlation between variables; that is, the closer the PCC to 1 or −1, the stronger the correlation. The closer the PCC to 0, the weaker the correlation. In the process of text readability measurement, the value range in Table 2 is usually used to judge the correlation strength between the two sequences.

### 4.3. Experimental Environment and Super Parameter Settings

The experimental environment and super parameter settings are shown Table 3. The laboratory is completed under Ubuntu system (Python 3.5 version), and other environment parameters are shown in Table 3.

In the setting of super parameters, it is unrealistic to find the learning rate that can make the convergence speed of loss function moderate and find the global optimal solution based on personal experience or multiple experiments, so the learning rate of the network model is set as the initial value, that is, the dynamic learning rate of 0.001, and the corresponding parameters are automatically updated during model training. A learning rate which is more suitable for the model can be found. In the convolution layer of the first level network of the hybrid network model, in order for the model to capture local information more comprehensively, such as phrase information with different lengths, we set the size of the convolution kernel to 3, 4, and 5; extract the corresponding features, respectively; and splice them into the total features.

Other hyperparameter settings are shown in Table 4.

### 4.4. Analysis of Experimental Results

#### 4.4.1. Comparison with CNN and LSTM Related Models

As shown in the experimental results in Table 5, we conducted experiments on various models related to CNN and LSTM on the gold standard data set WeeBit and compared them with the hybrid network model proposed in this paper.

Firstly, as we know, compared with the long short-term memory network, which only considers the following information: the bidirectional long short-term memory network can extract effective long-distance dependence and other information because it considers the context information. Therefore, CNN and BiLSTM are selected in the hybrid network model. Secondly, in theory, long short-term memory networks (including LSTM and BiLSTM) should be better at dealing with the task of sequence data input than convolutional neural network (CNN), but from the experimental results, the performance of long short-term memory network is slightly inferior to convolutional neural network model. The reason for this result may be that our network model takes the whole text sequence composed of word sequence as the input, and the length of the sequence is uncertain and long, which limits the performance of LSTM to a certain extent. Finally, in the hybrid network model, the final text representation can be calculated directly using the final state of LSTM or BiLSTM instead of the output of the intermediate state of the cyclic network. However, experiments show that it is better to retain the output of the intermediate state and connect the pooling layer. Moreover, we also need to properly consider the selection of the pooling layer connected after LSTM output. Considering the use of the attention mechanism layer in the pooling layer will get the best model effect and can achieve an accuracy (ACC) of 0.886 and a Pearson correlation coefficient (PCC) of 0.938 on the WeeBit data set.

#### 4.4.2. Comparison with the Existing Traditional Methods

As shown in Tables 6 and 7, we use the hybrid network model to do empirical research on WeeBit data set and Weekly Reader data set, respectively, and compare the experimental results with the results of existing model methods on the corresponding data set.

The experimental results show that the accuracy (ACC) of the proposed hybrid network model is 0.891 and the Pearson correlation coefficient is 0.932 on the WeeBit data set, while the accuracy (ACC) of 0.775 and Pearson correlation coefficient (PCC) of 0.836 are obtained on the Weekly Reader data set. It can be seen from the table that under the two measurement indices of accuracy and Pearson correlation, the performance of this hybrid network model is better than most traditional methods, but it is slightly inferior to the best model methods. In general, the hybrid network model has achieved competitive performance compared with traditional methods. In particular, it can automatically extract text readability related features, completely replace labor, liberate labor, and greatly improve the practicability of the model method in the task of text readability measurement.

## 5. Conclusions

Traditional text readability measurement methods have some fatal pain points. In the research process of text readability measurement, feature selection excessively depends on human experts, which limits the development of text readability measurement. There are a wide variety and a large number of existing features that measure text readability. It is more and more difficult to extract new features manually to improve the readability measurement performance, and even introduce redundant and irrelevant features to affect the readability measurement performance. To solve these problems, this paper proposes a hybrid network model for text readability measurement based on convolutional neural network, makes an empirical study on this method, and evaluates the performance of the model.

The proposed hybrid network model based on convolutional neural network has limitations or deficiencies in measuring text readability. Firstly, the hybrid network model regards the whole document as a sequence composed of one word. Due to the different length of the text, it will be filled with 0 in the process of processing the equal length input, which will introduce a lot of redundant information into the sequence features extracted by the network model, which will affect the performance of the model. Secondly, because the whole document is directly used as an input sequence, the factors that can affect the readability of the text contained in the sentence related information in the text (such as the logical structure and syntactic relationship between sentences) will be lost. Finally, because the network model takes the word sequence of the whole document as the input, the text will be relatively long theoretically, ranging from hundreds of words to thousands of words. In the process of processing such a long sequence, the gradient will disappear. With the continuous growth of the sequence length, some context information will be lost after long-distance information transmission. This limits the performance of long short-term memory networks. Future research will focus on how to overcome the limitations of hybrid network model and the construction of improved hybrid network model, such as hierarchical hybrid network model.

## Figures and Tables

**Figure 1:** CNN model structure.

**Table 1:** The details of Weekly Reader corpus and WeeBit corpus.

	Reading level	Applicable age	Number of chapters	Average number of sentences per text
Weekly Reader corpus	Level 2	7-8	633	23.45
	Level 3	8-9	795	23.22
	Level 4	9-10	805	29.17
	Senior	10–12	1316	31.22
WeeBit corpus	Level 2	7-8	641	23.01
	Level 3	8-9	791	23.45
	Level 4	9-10	822	29.23
	KS3	11–14	652	22.11
	GCSE	14–16	3600	28.22

**Table 2:** PCC value range and its correlation strength.

PCC value	Correlation strength
0–0.2	Very weak correlation or no correlation
0.2–0.4	Weak correlation
0.4–0.6	Moderate correlation
0.6–0.8	Strong correlation
0.8–1	Extremely strong correlation

**Table 3:** Experimental environment parameters.

Name	Parameter
Memory	15.6 G
Graphics	GeForce GTX 1080 Ti/PCLe/SSE2
Processor	Intel Core^TM^ i7-8700 CPU @ 3.7 GHz x 12

**Table 4:** Hyperparameter settings.

Hyperparameter	Introduction	Value
learning.rate	Initial value of learning rate	0.001
embedding.size	Word vector dimension	100
filter.size	Convolution kernel size	3,4,5
num.filter	Number of convolution kernels	200
Dropout	Dropout probability size	0.5
l2.reg.lambda	Size of L2 regularized lambda	0.0001
lstm.hidden	LSTM hidden layer size	100
batch.size	Batch size	100
max.length	Length of sequence	1538

**Table 5:** Comparison with CNN and LSTM related models.

Model	Accuracy	Pearson correlation coefficient
CNN	0.801	0.840
LSTM	0.711	0.744
BiLSTM	0.719	0.836
CNN-BiLSTM	0.831	0.892
CNN-BiLSTM-MoT	0.877	0.921
CNN-BiLSTM-ATT	0.886	0.938

**Table 6:** Comparison with existing traditional methods (on WeeBit data set).

Model	Accuracy	Pearson correlation coefficient
Model 1 [33]	0.929	—
Model 2 [34]	0.811	0.902
The proposed model	0.891	0.932

**Table 7:** Comparison with existing traditional methods (on Weekly Reader data set).

Model	Accuracy	Pearson correlation coefficient
Model 3 [30]	0.732	—
Model 4 [31]	0.628	—
Model 1 [33]	0.911	—
The proposed model	0.775	0.836

## Data Availability

The data set can be accessed upon request.
